RETRACTED

# Zinc sulfate contributes to promote telomere length extension via increasing telomerase gene expression, telomerase activity and change in the *TERT* gene promoter CpG island methylation status of human adipose-derived mesenchymal stem cells

**DOI:** 10.1371/journal.pone.0188052

**Published:** 2017-11-16

**Authors:** Raheleh Farahzadi, Ezzatollah Fathi, Seyed Alireza Mesbah-Namin, Nosratollah Zarghami

**Affiliations:** 1 Hematology and Oncology Research Center, Tabriz University of Medical Sciences, Tabriz, Iran; 2 Department of Clinical Biochemistry, Faculty of Medical Sciences, Tarbiat Modares University, Tehran, Iran; 3 Department of Clinical Sciences, Faculty of Veterinary Medicine, University of Tabriz, Tabriz, Iran; 4 Stem Cell Research Center, Tabriz University of Medical Sciences, Tabriz, Iran; 5 Department of Medical Biotechnology, Faculty of Advanced Medical Sciences, Tabriz University of Medical Sciences, Tabriz, Iran; University of Newcastle, UNITED KINGDOM

## Abstract

The use of mesenchymal stem cells (MSCs) for cell therapy and regenerative medicine has received widespread attention over the past few years, but their application can be complicated by factors such as reduction in proliferation potential, the senescent tendency of the MSCs upon expansion and their age-dependent decline in number and function. It was shown that all the mentioned features were accompanied by a reduction in telomerase activity and telomere shortening. Furthermore, the role of epigenetic changes in aging, especially changes in promoter methylation, was reported. In this study, MSCs were isolated from the adipose tissue with enzymatic digestion. In addition, immunocytochemistry staining and flow cytometric analysis were performed to investigate the cell-surface markers. In addition, alizarin red-S, sudan III, toluidine blue, and cresyl violet staining were performed to evaluate the multi-lineage differentiation of hADSCs. In order to improve the effective application of MSCs, these cells were treated with 1.5 × 10^−8^ and 2.99 × 10^−10^ M of ZnSO_4_ for 48 hours. The length of the absolute telomere, human telomerase reverse transcriptase (*hTERT*) gene expression, telomerase activity, the investigation of methylation status of the *hTERT* gene promoter and the percentage of senescent cells were analyzed with quantitative real-time PCR, PCR-ELISA TRAP assay, methylation specific PCR (MSP), and beta-galactosidase (SA-β-gal) staining, respectively. The results showed that the telomere length, the *hTERT* gene expression, and the telomerase activity had significantly increased. In addition, the percentage of senescent cells had significantly decreased and changes in the methylation status of the CpG islands in the *hTERT* promoter region under treatment with ZnSO_4_ were seen. In conclusion, it seems that ZnSO_4_ as a proper antioxidant could improve the aging-related features due to lengthening of the telomeres, increasing the telomerase gene expression, telomerase activity, decreasing aging, and changing the methylation status of *hTERT* promoter; it could potentially beneficial for enhancing the application of aged-MSCs.

RETRACTED

## Introduction

Telomeres are composed of long-hexamer (TTAGGG) repeats at the end of eukaryotic chromosomes [1]. This nucleoprotein structure prevents chromosome instability, replicative senescence, end-to-end fusions of chromosomes, accelerated aging, and cancer [2, 3]. During the process of cell division, as a result of the imperfect replication of linear chromosomes, telomeres are shortened; this is called ‘end-replication problem’. Although the detailed molecular mechanisms of aging are not fully understood, progressive telomere shortening is one of the molecular mechanisms underlying ageing as critically short telomeres trigger chromosome senescence and loss of cell viability [4, 5]. Telomerase, a ribonucleoprotein enzyme, which is composed of Telomerase Reverse Transcriptase (TERT), the Telomerase RNA Component (TERC) as the RNA template, and telomerase-associated proteins, is responsible for adding telomeric repeats to the ends of chromosomes [1]. In most human somatic cells (except for stem cells), the level of telomerase activity usually diminishes after birth [6]. In contrast, telomerase is highly expressed in human cancer cells, germ line and progenitor cells [7]. The role of telomerase in cancer and ageing, two complicated biological processes, has been implicated. To investigate the mechanisms involved in the regulation of telomerase and aging, therefore, leads to a bright horizon in the field of aging and related issues. The presence of a large CpG island with dense CG-rich content in the human *TERT* (*hTERT*) gene promoter suggests that DNA methylation may play a role in the regulation of the *hTERT* expression. Several studies indicated that the DNA methylation pattern of *hTERT* is inconsistent with the hypothesis that DNA methylation of promoter CpG islands is typically associated with gene silencing. In this context, Devereux et al. (1999) showed a strong correlation between *hTERT* expression and telomerase activity [8]. Also, this study demonstrated that *hTERT* promoter methylation is involved in the regulation of *hTERT* expression and telomerase activity, at least in some cells. In addition, another study by Guilleret et al. (2002) supported the positive correlation between telomerase activity, *hTERT* gene expression, and the methylation of the *hTERT* promoter [9]. The role of methylation in the *hTERT* promoter has been investigated by several studies [8, 10]; however, no obvious conclusion could be drawn, and the role of methylation in *hTERT* regulation remains unknown.

RETRACTED

Mesenchymal stem cells (MSCs) have attracted great interest because of their multilineage differentiation potential, self-renewal properties, and their possible use of cell and gene therapies [11–13]. Despite the aforementioned advantages of MSCs, the specified properties of MSCs are strongly affected by aging [14–16]. As a result, the use of MSCs from older donors is lower than younger donors, which restricts clinical applications such as regenerative medicine or cell therapy. Asumda et al. (2011) demonstrated the significant differences in the morphology, population size, proliferation, population-doubling time, and differentiation potential of the Bone marrow-derived Mesenchymal Stem Cells (BMSCs) of young rats in comparison to the bone marrow of old rats [17]. Aminizadeh et al. (2016) reported that telomere length in aged BMSCs was significantly lower than their young counterparts and they showed that the mRNA expression of *TERT* and *TERC* were significantly lower in aged subjects [18]. In addition, Flores et al. (2008) reported that telomere length was shorter in aged stem cells and this loss of telomere length may also have a role to play in the dysfunction of aged stem cells [19].

Based on the theories of aging, it is believed that aging is most probably caused by free radicals generated as by-products during normal metabolism. It is, therefore, crucial to maintain the proliferation and differentiation capacity of MSCs. The use of antioxidants to prevent cellular aging is important. The role of the element zinc as an antioxidant and an anti-inflammatory agent for many chronic diseases such as cancers, neurodegeneration, immunologic disorders, and the aging process has been shown [20]. In a previous study, Nemoto et al. (2000) reported that providing additional zinc in the cell-culture medium increases the telomerase activity [21]. In another study, Bao et al. (2013) demonstrated that a decrease in the concentration of intracellular zinc and the zinc-binding protein, metallothionein, in peripheral-blood mononuclear cells in older subjects are associated with a decrease in telomere length and percentage of cells with critically short telomeres [22]. In addition to the role of zinc ion in aging, its role in differentiation of MSCs has been shown. It is believed that Zn^+2^ supplementation stimulated osteoblast and osteoblast differentiated gene expression [23]. In this regard, Fathi and Farahzadi (2017) indicated that 0.432 μg/ml ZnSO4 induced the osteogenic differentiation of rat adipose tissue-derived MSCs via PKA, ERK1/2, and Wnt/β-catenin signaling pathways [24]. This induction resulted in an increase in the expression of osteogenic genes such as ALP, OCN, BMP2 and Runx2, ALP activity and calcium levels [24].

RETRACTED

However, it remains unclear whether ZnSO_4_ supplementation can increase the telomere length and change the methylation status in the *hTERT* gene promoter in hMSCs, and whether there exists a relationship between the telomere length and the hypomethylation or hypermethylation of CpG islands in the *hTERT* promoter region. Therefore, this study was carried out to investigate the effect of ZnSO_4_ on the telomere length, the *hTERT* gene expression, the telomerase activity, the percentage of senescent cells, and the methylation status of CpG islands in the *hTERT* promoter region in hMSCs.

## Materials and methods

### Reagents

All materials were purchased from Sigma-Aldrich (St. Louis, MO, USA), unless otherwise stated. All tissue culture plastic ware was from SPL Life Sciences (Pocheon, Korea). A comprehensive overview of methods that have been used in this paper was described as Fig 1.

**Fig 1:** Flow chart of an overview of the experimental procedures that have been done in this paper.

### Sampling

Adipose tissue samples were collected from the six normal women (45∼58 years old) after undergoing liposuction surgery performed at the Imam Reza Hospital, Tabriz University of Medical Sciences, Tabriz, Iran. All participants provide their written informed consent to participate in this study. This stage of the project was approved by the ethics committee of Tabriz University of Medical Sciences, Tabriz, Iran (registered number No.91/4-3/1).

### Isolation and cultivation of human adipose tissue-derived mesenchymal stem cells

The human adipose tissue-derived mesenchymal stem cells (hADSCs) were isolated as previously described in another paper by Farahzadi et al. (2016) [25]. At brief, the adipose tissues were washed with phosphate-buffered saline (PBS), minced to 1 mm^2^ pieces, and digested enzymatically for 30 minutes at 37°C, using 0.075% (w/v) collagenase type I (Invitrogen, UK). Collagenase activity was neutralized with fetal bovine serum (FBS) and centrifuged at 800×g for 5 minutes to obtain a pellet. The resulting pellet was re-suspended in a complete culture medium (Dulbecco’s modified Eagle’s Medium (DMEM) supplemented with 5% penicillin/streptomycin and 10% (v/v) FBS, and this pellet was added into a 24-wells plate followed by incubation at 37°C with 5% CO_2_ in a humidified environment for three days. The medium was replaced with a fresh medium every 3–4 days during cultivation. When the cells became confluent, they were trypsinized with 0.25% trypsin (Gibco, UK) and 1 mM EDTA (Invitrogen, UK), and then sub-cultured; hADSCs at Passage 3–6 were used in this study [26, 27].

RETRACTED

### Phenotypical characterization of human adipose tissue-derived mesenchymal stem cells

#### Immunocytochemistry staining

A total of 4 × 10^3^ cells were seeded in an 8-wells cell culture chamber slide. After one day of culture, the cells were washed with PBS and then fixed in 4% paraformaldehyde for 30–60 minutes at room temperature. After fixation, the cells were washed twice with PBS, and once with PBS and 1% BSA. The cells were incubated overnight at 4°C with a 1:100 dilution of mAbs against CD90, CD105, CD45, and CD56 (all from BD Biosciences, San José, CA) in PBS and 1% BSA. The cells were then washed with PBS and 1% BSA, and incubated with a 1:500 dilution of the biotin-conjugated mouse monoclonal IgG1 antibody against rats in PBS and 1% BSA for 1 hour. After washing with PBS, a 1:500 dilution of Streptavidin Alexa Fluor™ 488 conjugate (Molecular Probes, Eugene, OR) was added for 1 hour. The cells were washed three times with PBS and the nuclei were stained with 7.5 μM of propidium iodide (PI) for 15 minutes. After three washes with PBS, the fluorescent cells were visualized under the fluorescence microscope. The pluripotent capacities of the isolated hADSCs were confirmed with multilineage differentiation [28].

#### Flow-cytometric analysis

Approximately 10^6^ cells were washed twice with PBS containing 3% FBS (washing buffer) and were incubated with fluorescein isothiocyanate (FITC)-conjugated antibody CD31, CD34 and phycoerythrin (PE)–conjugated CD44, CD73 (BD Phar-mingen, San Diego, CA, USA) (1μg/10^6^cells) in washing buffer for 30 min on ice. hADSCs were washed with washing buffer again and FACSCalibur system (BD Biosciences, San Diego, CA) was used for characterization of hADSCs. Data were analyzed using with the FlowJo software (version 6.2).

#### In vitro multi-lineage differentiation of human adipose tissue-derived mesenchymal stem cells

hADSCs were grown to confluence and the multilineage differentiation of cells was induced in a complete culture medium containing one of the following four induction mediums as follow: (1) adipogenic differentiation medium: 0.5 mM 1-methyl-3 isobutylxanthine, 10 μg/ml insulin, 200 μM indomethacin and 1μM dexamethasone; (2) osteogenic differentiation medium: 0.05 mM L-ascorbic acid-2-phosphate, 10 mM b-glycerophosphate and 10 nM dexamethasone; (3) chondrogenic differentiation medium: ITS+1 Liquid Media Supplement (100x), 1.3 mM L-ascorbic 2-phosphate and 0.01 mM dexamethasone; (4) neurogenic differentiation medium: 200 ng/ml L-ascorbic acid-2-phosphates, 10 ng/ml GDNF, 20 ng/ml EGF and 20 ng/ml bFGF. After 14 days for neurogenic differentiation, and 21 days for adipogenic, osteogenic, and chondrogenic differentiation, the cells were fixed with 4% (v/v) paraformaldehyde for appropriate differentiation-specific staining: Sudan III (1% in 96% ethanol) for adipogenesis, alizarin red (2% in distilled water) for osteogenesis, toluidine blue (0.1% in distilled water) for chondrogenesis, and Cresyl violet (0.5% in 0.6% glacial acetic acid) for neurogenesis [24, 29–31].

RETRACTED

#### RNA extraction and reverse transcription (RT)-PCR analysis of multi-lineage differentiation-specific gene expression

Total RNA from the adipogenic, osteogenic, chondrogenic, and neurogenic differentiated cells was isolated using the Trizol reagent (Invitrogen, UK). The extracted cellular RNA was dissolved in diethyl phosphorocyanidate-treated water. After DNase treatment by the DNase I Amplification Grade Kit (Invitrogen, Paisley, Scotland), 2 μg RNA was used for the first strand of cDNA synthesis in a total volume of 20 μL according to the manufacturer’s guidelines. The regimen for RT-PCR was 15 minutes at 94°C, followed by the appropriate number of cycles of 1 minute at 94°C, 1 minute at the proper annealing temperature for each primer pair, and 1 minute at 72°C, with a final 10-minute extension at 72°C. The reaction mixtures for PCR included 20 ng of cDNA, TEMPase Hot Start 2x Master Mix І Blue (Ampliqon A/S, Denmark), and 0.5 μM of each antisense and sense primer as shown in Table 1. The amplified PCR products were analyzed by ethidium bromide staining after 1.5% agarose gel electrophoresis. The PCR primers were designed with the Oligo 7 primer design software [32–36].

**Table 1:** Primer sequences used for the RT-PCR assays.

No.	Gene	Primer pair sequence (5'-3')	Product length (bp)
NM_000478.5	ALP	ATGGGATGGGTGTCTCCACA CCACGAAGGGGAACTTGTC	108
NM_199173.5	OCN	GGCAGCGAGGTAGTGAAGA TCAGCCAACTCGTCACAGTC	131
NM_005036.4	PPAR-α	CAGAACAAGGAGGCGGAGGTC TTCAGGTCCAAGTTTGCGAAGC	119
NM_138711.3	PPAR-γ	GCCCTTTGGTGACTTTATGGA GCAGCAGGTTGTCTTGGATG	170
NM_001135.3	Aggrecan	TCGAGGACAGCGAGGCC TCGAGGGTGTAGCGTGTAGAGA	85
NM_001844.4	Collagene II	GGCAATAGCAGGTTCACGTACA CGATAACAGTCTTGCCCCACTT	79
NM_002506.2	NGF	GGACCCAATAACAGTTTTACC GAACAACATGGACATTACGC	81
NM_006617.1	Nestin	GAAGGTGAAGGGCAAATCTG CCTCTTCTTCCCATATTTCCTG	97
NM_002046.5	GAPDH	ATGGGGAAGGTGAAGGTCG GGGGTCATTGATGGCAACAATA	108

### Determining suitable concentration of ZnSO_4_ and cell proliferation by MTT assay

The MTT (3-(4, 5-dimethylthiazol-2-yl)-2, 5-diphenyl tetrazolium bromide) test was used to determine suitable concentration of ZnSO_4_. For this purpose, hADSCs were seeded into 96-wells culture plate at 4×10^3^ cells/wells. Cells incubated for 24h at 37°C in a humidified environment with 5% CO_2_ to grow the cells in a monolayer. ZnSO_4_ was added to the wells at final concentrations of 1.5×10^−5^–10^−11^ and 2.99×10^−7^–10^−13^ M. Control wells were prepared by addition of complete culture medium. Following incubation time (24, 48 and 72 h), the media was replaced with MTT dye solution (2 mg/ml) and then were incubated at 37°C in a 5% CO_2_ incubator for 4 h. After further incubation for 4 h, the MTT solution was removed and formazan crystals were dissolved in dimethyl sulfoxide (100 μL). The optical density of each well was measured in an ELISA reader at a wavelength of 570 nm [37, 38].

RETRACTED

### Calculation of human adipose tissue-derived mesenchymal stem cells population doubling time

To calculate the population doubling time (PDT), hADSCs from Passage 4 were counted and seeded into 6-wells plates at a density of 5×10^4^ cells/wells for about 24, 48, and 72 hours in the presence of 1.5×10^−8^ and 2.99×10^−10^ M ZnSO_4_. PDT was calculated according to the following formula: PDT = CT / PDN, where CT is the number of hours of the experimental period and PDN = log (N1 / N0) × 3.31. In this equation, N0 is the cell number at the beginning and N1 is the cell number at the end of the cell culture period. After the termination of the culture period (24, 48, and 72 hours), the cells were harvested and counted [38].

### Senescence-associated beta-galactosidase (SA-β-gal) staining

To determine the effect of ZnSO_4_ on the percentage of senescent cells, SA-β-gal staining was performed. hADSCs from passages 5, 7, 9, and 11 were harvested and treated with 1.5×10^−8^ and 2.99×10^−10^ M ZnSO_4_ in 5% CO_2_ at 37°C. Following incubation for 48 hours, the cells were washed twice with PBS, and were, respectively, fixed with 2% (vol. / vol.) formaldehyde and 0.2% (vol. / vol.) glutaraldehyde for 5 minutes at room temperature. After that, the cells were washed with PBS again and incubated with a fresh beta-galactosidase substrate staining solution (5 mM potassium ferricyanide, 5 mM potassium ferrocyanide, 40 mM citric acid/Na phosphate buffer, 2 mM magnesium chloride, 150 mM sodium chloride, containing 1 mg/ml 5-bromo-4-chloro-3-indolyl-D-**β**-galactosidase (X-gal) in distilled water) for overnight at 37°C in the conditional absence of CO_2_. The cells were thereafter washed twice with PBS and once with methanol, and allowed to air-dry for 30 minutes. Senescence cells were identified as blue-stained cells by standard-light microscopy and at least 100 stained cells were counted in 10 randomly selected fields per sample in order to determine the percentage of SA-**β**-gal-positive [39].

RETRACTED

### DNA isolation

hADSCs at Passage 4 were plated in 6-wells culture plates at a density of 15×10^4^ cells/wells with a complete medium. After 3 days, these cells were treated with various concentrations (1.5×10^−8^ and 2.99×10^-10^M) of ZnSO_4_ for up to 48 hours. Genomic DNA was isolated from the cells using the YTA Genomic DNA Extraction Mini Kit by following the manufacturer's instructions (Yektatajhiz Co., Iran). In brief, 300 ng of proteinase K were added to the cell pellet and were incubated for 30 minutes at 60°C. After incubation, 200 μl of ethanol (96~100%) was added, mixed thoroughly by pulse-vortexing, and carefully transferred from the sample mixture to the BG column. The mixture was centrifuged at 8000×g for 1 minute and washed with 500 μl of washing buffer by the centrifuge for 1 minute at 14000×g, and then, the flow-through was discarded. The BG column was placed near the clean tube and 30~50 μl of elution buffer or ddH_2_O (pH 7.5~9.0) was added to the membrane center of the BG column. The column was centrifuged for 2 minutes at 14000×g to elute the DNA and the DNA fragment was stored at 4°C until it was required for absolute telomere length measurement and bisulfite modification. The required amount of DNA for absolute telomere length measurement and bisulfite modification is 20 and 500 ng/μl, respectively [40].

### Standard curves and associated calculations for absolute telomere length

#### Oligomers (standards and primers) preparation for absolute telomere length measurement

All oligomers should be HPLC-purified and diluted in an appropriate volume of TE buffer or ddH_2_O and stored at −20°C until required. Working solutions of oligomers should be made fresh—the dilutions are stable at 4°C for up to 2 weeks. Oligomer sequences were reported by O’Callaghan and Fenech (2011) (Table 2) [41]. Changes in the amount of template that is present in each reaction can by affected by pipetting or a DNA quantification error.

**Table 2:** Sequences of primers used in *hTERT* gene expression, absolute telomere assay and methylation specific PCR.

Oligomer name	Primer pair sequence (5'-3')	PCR product size (bp)
**hTERT**	Fwd: CCGCCTGAGCTGTACTTTGT Rev: CAGGTGAGCCACGAACTGT PCR program: 2 min at 94°C, followed by 40 cycles, each at 94°C for 15 s and at 63°C for 1 min	234
**β-actin**	Fwd: AAACTGGAACGGTGAAGGTG Rev: TATAGAGAAGTGGGGTGGCT PCR program: 2 min at 94°C, followed by 40 cycles, each at 94°C for 15 s and at 63°C for 1 min	174
**Telomere standard**	(TTAGGG)14	84
**36B4 standard**	5'CAGCAAGTGGGAAGGTGTAATCCGTCTCCACAGACAAGGCCA GGACTCGTTTGTACCCGTTGATGATAGAATGGG 3'	75
**Telo**	Fwd: CGGTTTGTTTGGGTTTGGGTTTGGGTTTGGGTTTGGGTT Rev: GGCTTGCCTTACCCTTACCCTTACCCTTACCCTTACCCT	>76
**36B4**	Fwd: CAGCAAGTGGGAAGGTGTAATCC Rev: CCCATTCTATCATCAACGGGTACAA	75
**Unmethylated** **(13F and 4R)**	Fwd: GGATTTGTGGGTATAGATGT (bases −223 to −203) Rev: AACATAACCAACAACAACACCT (bases 115 to 135)	358
**Methylated** **(9F and 5R)**	Fwd: GGATTCGCGGGTATAGACGTT (bases −223 to −203) Rev: AACGTAACCAACGACAACACCT (bases 115 to 135)	358

RETRACTED

#### Telomere standard curve

A standard curve is created by the dilution of the known quantities of a synthesized 84-mer oligonucleotide (84 bp in length) containing only TTAGGG, repeated 14 times as shown in S1 Fig. The number of repeats in each standard is previously reported by O’Callaghan and Fenech (2011) [41]. For generating a standard curve, the serial dilutions of TEL STD A (10^−1^ [1.18 ×10^8^] through to 10^−6^ [1.18 × 10^3^] dilution) is performed.

#### Single copy gene (SCG) standard curve

SCG is used as a control for determining the genome copies per sample. 36B4, which encodes the acidic ribosomal phosphoprotein P0, was routinely used. Unlike the consistency of telomeric DNA sequence in mammals, the SCG will be different; a SCG standard curve and amplicon must thus be generated for each target species. The SCG amplification is crucial for the accuracy and reliability of the results generated in the aTL assay. The genome copy number per reaction is calculated by O’Callaghan and Fenech (2011) [41]. For generating a standard curve, the serial dilutions of SCG STD A (10^−1^ through to 10^−6^ dilution) is performed as shown in S2 Fig.

### Real-time PCR amplification for absolute telomere length

Real-time PCR was performed on the Corbett Rotor-Gene™ 6000 HRM (Corbett Research, Australia) in a total volume of 20 μL containing DNA (20 ng/μl), 0.1 μM of each primer, Power SYBR Green Master Mix (2x) (TaKaRa Ex Taq HS, Japan), and H_2_O. Thermal cycles (for both telomere and 36B4 amplicons) were performed in the following program: 5 minutes at 95°C, 40 cycles at 95°C for 15 seconds, 64°C for 60 seconds, followed by a melt curve. The data obtained from real-time PCR technique to measure the absolute telomere length were analyzed as kb/reaction and the genome copies/reaction for the telomere and the SCG, respectively, as previously described by O'Callaghan and Fenech (2011) [41].

### Processing and analyzing data for measuring the absolute telomere length

Real-time PCR data were analyzed as kb/reaction for telomere and as genome copies/reaction for SCG. The kb/reaction value was then used to calculate total telomere length in kb per human diploid genome. The telomere kb per reaction value is divided by diploid genome copy number to give a total telomere length in kb per human diploid genome. The obtained value can be further used to give a length per telomere by dividing by 92 which is the total number of telomeres on 23 pairs of chromosomes found in normal human cells [25, 41].

RETRACTED

### Methylation analysis by methylation-specific PCR (MSP) and sequencing

The bisulfite modification was performed with the EZ DNA Methylation-Gold™ Kit (Zymo Research, Germany, Catalog Nos. D5005 and D5006) according to the manufacturer's instructions. Following the bisulfite modification, MSP was performed with primers designed to amplify the methylated or unmethylated sequences in a part of the first exon of the *hTERT* promoter (up to 45 CpG sites extending from 500 bases upstream into the first exon of the *hTERT* promoter) as listed in Table 2. Sequences for all the primers have been previously reported by Devereux et al. (1999) [8]. The PCR mixtures contained 20 ng of modified DNA, 0.5 μM primers, and TEMPase Hot Start 2x Master Mix І Blue (Ampliqon A/S, Denmark). The amplification conditions were as follows: denaturation at 95°C for 5 minutes; 40 cycles of 95°C for 1 minute, 56.7°C (13F and 4R primers) and 59°C (9F and 5R primers) for 1 minute, and 72°C for 1 minute; and a final elongation step of 72°C for 4 minutes. Subsequently, the PCR products were electrophoresed on 1.5% agarose gels, and the bands were excised and purified on Qiagen columns (Qiagen Inc., Santa Clarita, CA). The products were then sequenced with a Macrogen Inc. (South Korea). Amplification primers were used as sequencing primers.

### Real-time PCR amplification for the *hTERT* expression

Real-time PCR to determine the *hTERT* gene expression was performed as previously described in detail by Farahzadi et al. (2016) [25]. In brief, after the treatment of hADSCs with 1.5×10^−8^ and 2.99×10^−10^ M ZnSO_4_ for 48 hours, cells were harvested and the cDNA was synthesized from the total mRNA by reverse transcription. Real-time PCR reactions were performed using the Corbett Rotor-Gene™ 6000 HRM (Corbett Research, Australia) in a total volume of 20 μl containing cDNA (40 ng/μl), 0.1 μM of each primer as shown in Table 2, the Power SYBR Green Master Mix (TaKaRa Ex Taq HS, Japan), and H_2_O. The data were analyzed using the 2^-ΔΔCT^ method to calculate the relative expression changes and the values expressed as fold-changes between the Ct value of *hTERT* (as the target gene) and the Ct value of *β-actin* (as the housekeeping gene) [42, 43].

### Telomerase activity assay

After the treatment of hADSCs with 1.5×10^−8^ and 2.99×10^−10^ M ZnSO_4_ for 48 hours, cells were lysed, total protein was extracted and then the protein concentration was measured with PicoDrop spectrophotometer (PICOPET01, UK). Relative telomerase activity of hADSCs in the presence and absence of ZnSO_4_ was assessed using the quantitative TeloTAGGG Telomerase PCR-ELISA kit (Roche Life Science, Mannheim, Germany), based on the manufacturerʼs protocol [18]. Briefly, cell extracts were incubated with biotin-labeled primers at 25°C, and the telomeric repeats added onto the ends of the primers were amplified by PCR. The PCR products were added to digoxigenin-labeled detection specific probes and following were allowed to bind to a streptavidin-coated 96-wells plate. Finally, the optical density of the blue color was measured at 450 nm by a STAT‑FAX 3200 ELISA reader (Awareness Technology, Inc., USA).

RETRACTED

### Quantitative real-time PCR measurements of osteocyte and adipocyte gene expression

Cells were cultured at a concentration of 30×10^4^ cells/wells in 6-wells plates containing an osteogenic induction medium for 48 hours in the presence and absence of 1.5×10^−8^ and 2.99×10^−10^ M ZnSO_4_. After termination of treatment of cells with ZnSO_4_, total RNA from the cells was isolated and cDNA synthesis was carried out. All PCR reactions were performed using the Corbett Rotor-Gene™ 6000 HRM (Corbett Research, Australia) in a total volume of 20 μL containing Power SYBR Green master mix (2x) (TaKaRa Ex Taq HS, Japan), Primer fwd (0.5 μM), Primer rev (0.5 μM), cDNA (30 ng/μl) and H_2_O. The mRNA expressions of target genes in the hADSCs included ALP, OCN, PPAR-α and PPAR-γ. GAPDH was selected as an endogenous housekeeping gene. The thermal cycling conditions were beginning denaturation step 5 min at 95°C, followed by 40 cycles, each denaturation at 95°C for 10 s, annealing at 59°C (ALP, OCN and PPAR-γ) or 62°C (PPAR-α) for 15 s and extension at 72°C for 20 s. Fluorescence data was analysed as explained above. Also, primers were designed using Oligo 7 v.7.52 software (Molecular Biology Insights, Inc, USA) and the sequences for each primer are presented in Table 1.

### Statistical analysis

The results were analyzed using the software program Graph Pad Prism version 6.01. The results were expressed as the means ± standard error (SE). We used one-way and two-way ANOVA followed by Dunnett’s post hoc test to determine the significant difference among groups. Also, for quantitative real-time RT-PCR analysis, the REST 2009 software (Qiagen) was used. Statistical significance was determined at p<0.05. All experimental procedures were repeated for three times.

## Results

### Phenotypical characterization of human adipose tissue-derived mesenchymal stem cells

Fig 2A showed that the hADSCs were spindle-shaped cells, both as scattered individuals and in small colonies; hADSCs had the capacity to adhere to the tissue-culture plastic flasks. Phenotypical characterization was performed by the immunocytochemistry for CD90, CD105, CD45, and CD56 as well as by flow cytometry for CD73, CD44, CD31, and CD34. Immunocytochemistry images revealed that the cultured cells were consistently positive for CD90 (B) and CD105 (C), and negative for CD45 (D) and CD56 (E) (Fig 2B–2E). Also, the hADSCs were consistently positive for CD73 (93.1%) and CD44 (80.2%), and negative for hematopoietic cell lineage-specific antigens, such as CD31 (0.02%) and CD34 (0.03%) (Fig 3).

RETRACTED

**Fig 2:** (A) Spindle-shaped morphology of hADSCs 7 days after seeding. Immunocytochemistry staining for the expression of hADSCs cell markers. (B) CD 90, (C) CD 105, (D) CD 45, and (E) CD 56. Nuclei were labeled with propidium iodide (PI) (orange) (bar = 40X).

**Fig 3:** The expression of the surface epitopes of hADSCs as analyzed by flow cytometry. Each antibody was tested individually and the isotopes controls were used as the negative control in this experiment; the ADSCs were positive for CD44 (80.2%) and CD73 (93.1%), and negative for CD31 (0.02%) and CD34 (0.03%). For CD44 and CD73, the isotype control was mouse IgG2b and for CD31 and CD34, the isotype control was mouse IgG1.

### Multilineage differentiation of human adipose tissue-derived mesenchymal stem cells to osteocyte, adipocyte, chondrocyte, and neurons lineage

Following osteogenic differentiation, the extracellular calcium matrix was stained with alizarin red. After the aforementioned staining, the redness of the nodules indicated the presence of mineralized compartments as a result of osteogenic treatment (Fig 4A). The gene expression of ALP and OCN as osteocyte-specific genes was confirmed with RT-PCR (Fig 4E). For adipogenesis confirmation of hADSCs, lipid droplets were stained with Sudan III (Fig 4B). The expressions of PPAR-α and PPAR-γ as adipocyte-specific genes were detected by RT-PCR analysis (Fig 4F). At the end of chondrogenic differentiation, the aggregates of aggrecan as key molecules within the cartilage matrix were stained with Toluidine blue (Fig 4C). RT-PCR analysis was shown the expression of Aggrecan and Collagene II (Fig 4G). After neural induction, the neuronal differentiation was determined by Cresyl violet by the positive staining of Nissl bodies. Nissl bodies appear dark black-violet with the background remaining almost colorless (Fig 4D). RT-PCR analysis identified the expression of NGF and nestin as neural markers in the treated cells (Fig 4H).

RETRACTED

**Fig 4:** In vitro multilineage differentiation of hADSCs. (A) Osteogenic differentiation and alizarin red staining of mineralized cell aggregates; (E) Detection of the two bone specific genes (ALP and OCN) by RT-PCR method (B) Generation of lipid vacuoles after adipogenesis; (F) Expression of PPAR-α and PPAR-γ as fat-specific genes; (C) After chondrogenesis of hADSCs, proteoglycan aggregates stain with toluidine blue; (G) RT-PCR analysis of aggrecan and collagen II as chondrocyte-specific genes; (D) The neuronal cells differentiated from hADSCs show extensive somata-associated accumulations of Nissl bodies stained dark black-violet; (H) Expression of nestin and NGF as neural-specific genes (bar = 40X).

### Cell proliferation activity and PDT of human adipose tissue-derived mesenchymal stem cells

To determine the range of physiological concentrations of ZnSO_4_ for experimental conditions, hADSCs were exposed to various concentrations of ZnSO_4_ (1.5 × 10−5–10^−11^ and 2.99 × 10−7–10^−13^ M) for a total of 24, 48, and 72 hours. As shown by the MTT assay (Fig 5A), ZnSO_4_ had no significant impact at concentrations between 1.5 × 10−5–10^−7^, 1.5 × 10−9–10^−11^, 2.99 × 10−7–10^−9^, and 2.99 × 10^−11^ − 10^−13^ M, but at concentrations of 1.5 × 10^−8^ and 2.99 × 10^−10^ M, a significant proliferation effect was seen (*P < 0.05). Therefore, at concentrations of 1.5 × 10^−8^ and 2.99 × 10^−10^ M, ZnSO_4_ was used in a complete culture medium to treat the cells.

**Fig 5:** **(A and B) Effect of various concentrations of ZnSO**_**4**_ **on the proliferation of hADSCs.** Cells were cultured at a density of 2 × 10^3^ cells/wells with various concentrations of ZnSO_4_ for 24, 48, and 72 hours, and their viability was measured by a MTT assay. The MTT dye solution was added when the hADSCs were cultured for 24, 48, and 72 hours, respectively. After 4 hours of incubation, the culture medium was removed, DMSO was added, and the optical density of each well was measured at a wavelength of 570 nm (*P < 0.05 compared with control group). The results of Fig 5A in the X axis based on the serial dilution. **(C) Population doubling time (PDT) of hADSCs after treatment with 1.5×10**^**−8**^ **and 2.99×10**^**−10**^ **M ZnSO**_**4**_ **in comparison to the control.** Cells were seeded at a density of 5×10^4^ cells/wells for about 24, 48, and 72 hours in the presence of 1.5×10^−8^ and 2.99×10^−10^ M ZnSO4. PDT was calculated according to the following formula: PDT = CT / PDN. The results indicated significantly short PDTs of ZnSO_4_-treated cells in comparison to that of untreated cells (*P < 0.05 compared with control group). To calculate cell proliferation and PDT for each treatment with ZnSO_4_, 3 wells of culture plate was considered, this procedure was repeated for three times. Data represent as the means ± SE from three independent biological experiments. Two-way ANOVA followed by Dunnett’s post hoc test was used in all parts of Fig 5.

RETRACTED

As shown in Fig 5B, the PDT value was 17.5 hours for control group of cells, whereas this value was recorded as 17.63 hours, 10.98 hours, and 16.10 hours after treatment with 1.5×10^−8^ M ZnSO_4_ for 24, 48, and 72 hours, respectively. In addition, the PDT value was recorded as 21.71 hours, 16.06 hours, and 19.98 hours after treatment with 2.99×10^−10^ M ZnSO_4_ for 24, 48, and 72 hours, respectively. Among these values, 10.98 hours and 16.06 hours were significantly different in comparison to control (*P < 0.05).

### Senescence-associated beta-galactosidase (SA-β-gal) staining

The amount of senescent hADSCs treated with various concentrations (1.5 × 10^−8^ and 2.99 × 10^−10^M) of ZnSO_4_ for up to 48 hours was investigated by the SA-**β**-galactosidase staining method. SA- **β**-gal stained cells first appeared in Passage 5 and increased in Passages 7, 8, and 9. The senescent percentages of cells were indicated in Fig 6. As shown in Fig 6A, 1.5×10^−8^ and 2.99×10^−10^ M ZnSO_4_ caused a reduction in the number of stained cells in Passages 5, 7, 9, and 11 (P < 0.001).

**Fig 6:** (A) The presence of senescent cells in different passage cultures. Senescent cells were first observed in Passage 5 and their number was increased as the passage number increased. Meanwhile, the treated of hADSCs for 48 hours in the presence of 1.5 × 10^−8^ and 2.99 × 10^−10^ M ZnSO_4_ cause a decrease in the number of stained cells (**P < 0.01 and *** P < 0.001 compared with control group). To count senescent cells for each treatment with ZnSO_4_, 3 wells of culture plate was considered, this procedure was repeated for three times. Data represent as the means ± SE from three independent biological experiments. Two-way ANOVA followed by Dunnett’s post hoc test was used to determine the significant difference among groups. (B) and (C) were included as a positive and negative controls for SA-**β**-galactosidase staining, respectively.

### The effect of ZnSO_4_ on absolute telomere length

Absolute telomere length measurement was evaluated using real-time PCR after 48 h treatment of hADSCs with 1.5×10^−8^ and 2.99×10^−10^ M ZnSO_4_. As shown in Fig 7, absolute telomere length increased in the presence of 1.5×10^−8^ M (6.53 Kbp) and 2.99×10^−10^ M ZnSO_4_ (4.27 Kbp) compared to the control group (3.89 Kbp). This increase just significant at concentration of 1.5×10^−8^ M ZnSO_4_ (**p<0.01).

RETRACTED

**Fig 7:** Absolute telomere length measurement of hADSCs in the presence of different concentration of ZnSO_4_ for 48 hours of incubation. Cells were seeded at a density of 5×10^4^ cells/wells for about 48 hours in the presence of 1.5×10^−8^ and 2.99×10^−10^ M ZnSO_4_. Following, Genomic DNA was isolated, telomere and single copy gene standard curve was created. Real-time PCR technique was used to measure the absolute telomere length. The data were analyzed as kb/reaction and the genome copies/reaction for the telomere and the SCG. As described in results section, 1.5×10^−8^ M ZnSO_4_ were significantly increased the telomere length of hADSCs (**P<0.01 compared with control group), this procedure was repeated for three times. Data represent as the means ± SE from three independent biological experiments. One-way ANOVA followed by Dunnett’s post hoc test was used to determine the significant difference among groups.

### Determination of CpG Islands in the *TERT* gene promoter

At first, the *hTERT* gene promoter sequence was prepared from the NCBI database. Data from this database indicates that the promoter of this gene occurs in the Gene Bank with the code AF097365.1 and has 4,355 base pairs. In order to determine the CpG Islands in this sequence, online CpG Islands prediction software (http://www.urogene.org) was thereafter used. As shown in S3 Fig, in this sequence, there are several CpG Islands that have been identified possessing a light blue color. The intended CpG Islands were, therefore, elected for the nucleotides 3515 to 4298. In addition, Fig 8 shows a schematic representation of the 45 sites susceptible to methylation in the *hTERT* gene promoter.

**Fig 8:** The schematic figure for showing the 45 CpG sites of the *hTERT* promoter.

### *hTERT* promoter methylation assessment

Extending the 500 bases upstream into the first exon of the *hTERT* promoter, from the bases −223 to −203, and the bases 115 to 135, 45 CpG sites were studied. The results of the *hTERT* promoter methylation indicated that the mentioned region of this gene (from the bases −223 to −203 and the bases 115 to 135) is differentially methylated and unmethylated in the treated group with ZnSO_4_ in comparison to the control group. In both groups, in the presence and absence of 1.5×10^−8^ and 2.99×10^−10^ M ZnSO_4_, the MSP sequencing revealed the unmethylated and methylated CpG sites. Among the 45 sites of these CpG islands, 5 sites were converted from unmethylated to methylated and 9 sites were converted from unmethylated to methylated. In addition, the state of 7 unmethylated sites and 10 methylated sites remained unchanged. Due to incongruent results obtained from three replications of this experiment the other sites has not been determined (Figs 9 and 10, Table 3).

RETRACTED

**Fig 9:** The results of the original sequence alignment of the *hTERT* promoter region from 500 bases upstream into the first exon, sequence without treatment, and treated sequences with various concentrations of ZnSO4. The first sequence from the top is the original sequence (main sequence) that was obtained from the NCBI database; the second, third, and fourth sequence from the top are related to the samples without treatment (control), treated with 1.5×10^−8^ M, and 2.99×10^−10^ M ZnSO_4_, respectively. The CpG sites are shown by the pink arrow.

**Fig 10:** The sequence of 500 bases upstream into the first exon of the *hTERT* promoter and its transcription factor binding sites. The sequence from bases −223 to −203, and bases 115 to 135 of the *hTERT* promoter has been shown in the 5′ to 3′ direction, spanning 358 nucleotides, containing 45 CpG sites. The transcription factors whose binding sites have been determined using the online TFBIND INPUT database are presented here in italics.

**Table 3:** Methylation of the *hTERT* promoter region from 500 bases upstream into the first exon before and after treatment with various concentrations of ZnSO_4_. The CpG sites are numbered from 1–45, CpG sites are indicated as follows: methylation (M); unmethylation (U); not determined (-).

**Number of CpG sites**	**1**	**2**	**3**	**4**	**5**	**6**	**7**	**8**	**9**	**10**	**11**	**12**	**13**	**14**	**15**
**Control without ZnSO**_**4**_ **treatment**	**U**	**U**	**U**	**M**	**M**	**M**	**U**	**M**	**U**	**U**	**U**	**M**	**-**	**-**	**U**
**Treatment with 1.5×10**^**−8**^ **M ZnSO**_**4**_	**M**	**-**	**-**	**-**	**U**	**U**	**U**	**M**	**U**	**-**	**U**	**U**	**-**	**-**	**M**
**Treatment with 2.99×10**^**−10**^ **M ZnSO**_**4**_	**-**	**-**	**-**	**-**	**U**	**U**	**U**	**M**	**U**	**-**	**U**	**U**	**-**	**-**	**M**
**Number of CpG sites**	**16**	**17**	**18**	**19**	**20**	**21**	**22**	**23**	**24**	**25**	**26**	**27**	**28**	**29**	**30**
**Control without ZnSO**_**4**_ **treatment**	**-**	**-**	**M**	**M**	**M**	**U**	**U**	**M**	**U**	**-**	**U**	**-**	**-**	**U**	**M**
**Treatment with 1.5×10**^**−8**^ **M ZnSO**_**4**_	**-**	**-**	**U**	**U**	**M**	**M**	**M**	**M**	**U**	**-**	**U**	**-**	**M**	**U**	**M**
**Treatment with 2.99×10**^**−10**^ **M ZnSO**_**4**_	**-**	**-**	**U**	**U**	**M**	**M**	**M**	**M**	**U**	**-**	**U**	**-**	**-**	**U**	**U**
**Number of CpG sites**	**31**	**32**	**33**	**34**	**35**	**36**	**37**	**38**	**39**	**40**	**41**	**42**	**43**	**44**	**45**
**Control without ZnSO**_**4**_ **treatment**	**M**	**M**	**M**	**M**	**-**	**M**	**U**	**M**	**U**	**-**	**M**	**M**	**M**	**M**	**M**
**Treatment with 1.5×10**^**−8**^ **ZnSO**_**4**_	**M**	**M**	**M**	**M**	**U**	**M**	**M**	**M**	**U**	**-**	**M**	**U**	**U**	**M**	**M**
**Treatment with 2.99×10**^**−10**^ **M ZnSO**_**4**_	**M**	**U**	**M**	**-**	**U**	**M**	**M**	**U**	**U**	**U**	**M**	**U**	**U**	**M**	**M**

RETRACTED

### The effect of ZnSO_4_ on the *hTERT* gene expression

Real-time PCR for the detection of the *hTERT* expression in ADSCs was carried out after 48 hours of culture in 1.5×10^−8^ and 2.99×10^−10^ M ZnSO_4_. As shown in Fig 11, the expression of *hTERT* gene was 2.39 and 1.13-fold higher in the presence of 1.5×10^−8^ and 2.99×10^−10^ M ZnSO_4,_ respectively than control group. However, this increase is only significant at 1.5×10^−8^ M ZnSO_4_ compared to the control group (*P<0.05).

**Fig 11:** Relative *hTERT* gene expression levels of hADSCs in the presence of ZnSO_4_ for 48 hours of incubation. Cells were seeded at a density of 1.5×10^3^ cells/wells for about 48 hours in the presence of 1.5×10^−8^ and 2.99×10^−10^ M ZnSO_4_. Following, total RNA was isolated and was subjected to Real-time PCR Relative mRNA level of *hTERT* in the presence of 1.5×10^−8^ and 2.99×10^−10^ M ZnSO_4_. As described in results section, 1.5×10^−8^ M ZnSO_4_ was significantly increased the *hTERT* gene expression of hADSCs (*P<0.05 compared with control group). This procedure was repeated for three times. Data represent as the means ± SE from three independent biological experiments. One-way ANOVA followed by Dunnett’s post hoc test was used to determine the significant difference among groups.

### The effect of ZnSO_4_ on telomerase activity

PCR-ELISA TRAP assay method was used to assess the telomerase activity in ZnSO_4_-treated and untreated cells. As shown in Fig 12, the telomerase activity was 1.77 and 1.40-fold higher in the presence of 1.5×10^−8^ and 2.99×10^−10^ M ZnSO_4,_ respectively than control group. However, this increase is only significant at 1.5×10^−8^ M ZnSO_4_ compared to the control group (*P<0.05).

**Fig 12:** Relative telomerase activity measurement of hADSCs in the presence of different concentration of ZnSO_4_ for 48 hours of incubation as detected by the PCR-ELISA TRAP assay. Cells were seeded at a density of 5×10^4^ cells/wells for about 48 hours in the presence of 1.5×10^−8^ and 2.99×10^−10^ M ZnSO_4_. Following, cells were lysed and protein were extracted from each sample. Relative telomerase activity was assessed in protein extracts by Telomerase PCR-ELISA kit. Heat inactivated cell extract served as the negative control. As described in results section, 1.5×10^−8^ M ZnSO_4_ was significantly increased the relative telomerase activity of hADSCs (*P<0.05 compared with control group). This procedure was repeated for three times. Data represent as the means ± SE from three independent biological experiments. One-way ANOVA followed by Dunnett’s post hoc test was used to determine the significant difference among groups.

RETRACTED

### The effect of ZnSO_4_ on osteocyte and adipocyte mRNA gene expression

To further investigate the effects of ZnSO_4_ on multi-lineage differentiation of hADSCs, quantitative Real-time PCR was used for the detection of ALP, OCN gene expression as osteogenic markers and PPAR-α and PPAR-γ gene expression as adipogenic markers. As shown in Fig 13, in the presence of 1.5×10^−8^ and 2.99×10^−10^ M ZnSO_4_, the expression of ALP, OCN, PPAR-α and PPAR-γ genes was significantly increased as compared with control group (p<0.05).

**Fig 13:** **ZnSO**_**4**_ **effect on (A) ALP, (B) OCN, (C) PPAR-α and (D) PPAR-γ mRNA expression in hADSCs.** Cells were cultured in 6-wells plates at a concentration of 30 × 10^4^ cells /wells. RNA was extracted from cultured hADSCs in the presence and absence of 1.5×10^−8^ and 2.99×10^−10^ M ZnSO_4_ as described in materials and methods section and was subjected to Real-time PCR assay (*P<0.05 compared with control group). This procedure was repeated for three times. Data represent as the means ± SE from three independent biological experiments. One-way ANOVA followed by Dunnett’s post hoc test was used to determine the significant difference among groups.

## Discussion

Aging is one of the most important factors in reducing the clinical application of MSCs in cell therapy and regenerative medicine [44]. Aging is an inherently complex process that is manifested within an organism at the molecular and cellular levels. Telomere shortening, the reduction of the *hTERT* expression, and a decrease in telomerase activity as well as changes in the *hTERT* gene promoter methylation cause replicative senescence or cell death [6]. It seems that gene expression regulation may be directly involved in the differentiation potential and aging of stem cells [45]. Böcker et al. (2008) reported that *hTERT* over-expression could prevent the senescence of human MSCs, and the cells showed significantly higher and unlimited proliferation capacities [46]. In another study, Aminizadeh et al. (2016) showed the positive correlation between the *TERT* gene expression, the telomere length, and the telomerase activity in aged-bone marrow stromal cells in the presence of glutathione monoethyl ester [18]. The correlation between free radical production and its impact on telomere and telomerase as biomarkers of aging has attracted considerable attention towards the cell transplantation approach [47]. Finding methods such as the use of antioxidant to overcome the free radical production and aging of cells will, therefore, significantly assist cell therapy. Zinc as an antioxidant agent that has a crucial role in oxidative stress with efficient contributions in the free-radical scavenging activity [22, 48]. Zinc functions as an antioxidant and its function can be identified in several mechanisms such as in the inhibition of NADPH oxidase and the decrease of the Reactive Oxigene Species (ROS) generation, as a co-factor of the superoxide dismutase (SOD) enzyme, as a catalyst in the dismutation of ^•^O_2_^−^ to H_2_O_2,_ in competition with Fe^2+^ and Cu^2+^ ions for binding to cell membranes and protein, and inhibiting the production of ^•^OH from H_2_O_2._ Furthermore, zinc has a role to play in the induction of the generation of metallothionein as an excellent scavenger of ^•^OH, which is one of the most effective mechanisms [20]. In addition, zinc increases the activation of antioxidant molecules, proteins, and enzymes such as glutathione, catalase, and SOD; it reduces the activity of oxidant enzymes such as NADPH oxidase and nitric acid synthase, and inhibits the lipid peroxidation products. Although the essentiality of the zinc ion (Zn^+2^) as an antioxidant and an anti-inflammatory agent in aging and age-related disease have been reported, the effect of Zn^+2^ on telomere as the guardian of the chromosome in aging, the *hTERT* gene expression and in the methylation status of *hTERT* gene promoter as well as the epigenetic mechanisms involved in aging are yet to be reported, and their mechanism of action is still unknown. The results obtained by Nemoto et al. (2000) provides the first evidence for metals, especially Zn^+2^, to be able to modulate telomerase in cancer cells by inducing an enhancement of its activity [21]. Contrary to the results of Nemoto et al., in another study, Ren et al. (2007) reported that zinc phthalocyanine (ZnPc) had the ability to inhibit telomerase activity [49]. Although the underlying mechanism remains unclear, a few studies have been published in relation to the effective mechanisms of zinc’s effect on telomeres, which can be effective in finding the fundamental mechanism. In a study, Ren et al. (2007) reported that octacationic ZnPc could induce intramolecular G-quadruplex telomeric structure transition from the anti-parallel to the parallel form, and it could induce the parallel structure formation in the cation-deficient condition [49]. Liu et al. (2004) showed that 80 μm/L ZnSO_4_ helps to maintain and shorten the telomere length of the hepatocytes L-02 and the hepatoma cells SMMC-7721, respectively [50]. They showed that the mechanism might be related to the inhibition of telomerase activity in the SMMC-7721 cells. This might also be the result of the activation of the p53 protein, a zinc-binding transcription factor that becomes active in response to multiple forms of stress and controls proliferation, survival, DNA repair, and the differentiation of cells. Therefore, the supplementation of zinc could affect the transcription of DNA and telomere length by the activation of the p53 in hepatoma cells [50]. In the present study, 1.5×10^−8^ and 2.99×10^−10^ M was used as the final concentration of ZnSO_4_. To determine a suitable range for Zn^+2^ under this study's experimental conditions, the MTT assay was used to evaluate cell viability. In this study, it was found that ZnSO_4_ had no impact on the viability of the cells between 1.5 × 10^−5^ − 10^−7^, 1.5×10^−9^ − 10^−11^, 2.99×10^−7^ − 10^−9^, and 2.99×10^−11^ − 10^−13^ M. To explore the mechanism of ZnSO_4_ on telomere length, the *hTERT* gene expression, the telomerase activity, the methylation status of *hTERT* gene promoter and the percentages of senescent cells, real-time PCR, PCR-ELISA TRAP assay, MSP, and senescence-associated SA-β-gal staining were respectively performed. As observable from the results, the percentage of the senescent cells significantly decreased in the ZnSO_4_-treated ADSCs in comparison to untreated cells. In addition, the telomere length as well as the *hTERT* gene expression and the telomerase activity were significantly increased in the presence of 1.5 × 10^−8^ M ZnSO_4_ by more than 1.67, 2.39 and 1.77 fold in comparison to the control group, respectively. In this study, methylation patterns of the CpG islands in the promoter regions of the *hTERT* gene was seen as follow: among the 45 sites of CpG into the first exon of the *hTERT* promoter, 5 sites were converted from unmethylation to methylation, and 9 sites were converted from methylation to unmethylation. In the other words, a switch from the unmethylated to the methylated 4 CpG islands sites No. 15, 21, 22, and 37, a switch from the methylated to the unmethylated 5 CpG islands sites No. 5, 6, 12, 18 and 19 and the remaining 9 CpG islands sites (8, 20, 23, 31, 33, 36, 41, 44, and 45) in the methylation status in the presence of ZnSO_4_ can be used as important evidence for the correlation of the *hTERT* promoter methylation/unmethylation status and the regulation of the *hTERT* gene expression.

RETRACTED

The results of this study indicated that there is a good relationship between *hTERT* gene expression, telomerase activity and telomere length in the presence of 1.5 × 10^−8^ M ZnSO_4_. In addition to variations in telomere length, *hTERT* gene expression and telomerase activity in the presence of 1.5 × 10^−8^ M ZnSO_4_, the results obtained from gene promoter methylation analysis under treatment with 1.5×10^−8^ and 2.99×10^−10^ M ZnSO_4_ indicates similar results, except for three regions 30, 32, and 38, which are provided in the Table 3. *hTERT* gene promoter methylation results are in contrast to the results obtained from extent of *hTERT* gene expression, telomerase activity and telomere length in the presence of two different concentrations of ZnSO_4_. Since the telomerase activity is tightly regulated by the expression of the *hTERT* gene [51], a claim for the association of the telomerase activity and the methylation of the *hTERT* promoter can be put forward. Nevertheless, the regulation and the stabilization of the telomere length is complex, and appears to involve several mechanisms [8]. The role of methylation of the promoter region of *hTERT* for regulation of the *hTERT* expression, the telomerase activity, and the telomere maintenance have been investigated; however, no obvious conclusion could be drawn, and the role of methylation in *hTERT* regulation remains unknown. [52]. Some studies have reported a direct relationship between *hTERT* promoter methylation and *hTERT* gene expression, telomerase activity and telomere length and some others have demonstrated the lack of correlation between them [8, 53]. The relationship between methylation status of *hTERT* promoter and 3 parameters (*hTERT* gene expression, telomerase activity and telomere length) depends on the type of cells (including normal, immortalized, and cancer cell lines from various tissues). In one study, Devereux, et al. (1999) indicated that methylation of either specific CpG sites or groups of CpG sites did not necessarily correlate with *hTERT* gene expression in some cell lines [8]. On the other hand, it is known that some cells maintain their telomeres by telomerase-independent mechanisms; thus, CpG methylation may be involved in the regulation of *hTERT* expression and telomerase activity in some cells or tissue types, but not others [53]. Several studies have reported the correlation between methylation status of *hTERT* promoter and the *hTERT* expression. The results obtained in the study of Bechter et al. (2002) indicated that CpG island methylation of the *hTERT* promoter played a role in regulating *hTERT* gene expression in patients with B-cell chronic lymphocytic leukemia [54]. In a study by Guilleret and Benhattar (2003), a positive correlation between the hypermethylation of the *hTERT* promoter and gene activation was demonstrated; the demethylation of the *hTERT* promoter allowed a reduction of the *hTERT* expression and vice versa [55]. This correlation in the methylation status of the *hTERT* promoter was opposite to the general model of DNA methylation. In our study, there was no common methylation pattern that correlated with *hTERT* gene expression, telomerase activity and telomere length among two treated cells with 1.5×10^−8^ and 2.99×10^−10^ M ZnSO_4._ Although the *hTERT* gene expression from the methylated promoter suggests that CpG island methylation is not a general mechanism of down-regulation for this gene, it may play a role in the regulation of *hTERT* expression in specific cell types and/or at some stage of development or carcinogenesis. We propose to provide evidence for a possible role for DNA methylation in the regulation of *hTERT* gene expression; subsequently, telomerase activity and telomere length in the presence of different concentrations of ZnSO_4_, the effect of ZnSO_4_ on the cells which lacked *hTERT* gene expression and exhibited complete methylation of the *hTERT* promoter, in the presence or absence of the demethylating agent 5-AZC to be done in another experimental research in the future. Our findings suggest that *hTERT* gene expression, telomerase activity and telomere length in the presence of 1.5×10^−8^ and 2.99×10^−10^ M ZnSO_4_ is complex and appears to involve both methylation-dependent and methylation-independent mechanisms. In conclusion, the results of this study showed, the lack of correlations between *hTERT* gene expression, telomerase activity and telomere length with the methylation status of the *hTERT* gene promoter in the presence of 1.5×10^−8^ and 2.99×10^−10^ M ZnSO_4_.

RETRACTED

In addition to the role of *hTERT* gene promoter methylation status in the regulation of gene expression, the presence of various transcriptional factors and transcriptional binding motifs indicates that regulation of gene expression reflects a rather complex mechanism that is not solely dependent on methylation [54]. Previous studies have shown that the 5'-*hTERT* regulatory region contains numerous binding sites for transcription factors [56]. As reported in studies, methylated CpG islands sites may directly inhibit the binding of transcription activator factors of *hTERT*, such as c-Myc, AP2, SP1 etc [57–59]. However, non-methylated sites may be a site for attachment of activator factors of hTERT transcription, thereby preventing attachment of transcription inhibitors [58].

As can be seen in Fig 10, different transcription factors can attach to CpG sites in the region of *hTERT* gene promoter. In order to recognize the type of attached factors, online TFBIND INPUT database has been used. Note that the sequence presented to this database has been the main sequence of *hTERT* gene promoter without treatment with zinc sulfate. However, it should be noted that the mentioned transcription factors may cause increase or decrease of the extent of *hTERT* gene expression by either binding or not non-binding to these sites given the methylation or non-methylation of CpG sites in the presence of ZnSO_4_. Considering the change in the status of methylation of CpG sites No. 5, 6, 12, 18, and 19 from methylated to non-methylated state in the presence of ZnSO_4_, it is expected that activator transcription factors including AP2, SP1 and B be able to attach to the non-methylated sites and prevent attachment of inhibiting transcription factors such as E2F and USF to non-methylated CpG regions [60–63]. Opposite of the mentioned state would occur regarding altered status of methylation from non-methylated to methylated [58]. According to the results of this study, it could thus be claimed that ZnSO_4_ with a changing methylation status of CpG islands causes the binding of transcription factors as activators or suppressors of the *hTERT* transcription and maybe cause the regulation of the *hTERT* gene expression.

RETRACTED

Although changing the methylation patterns at certain CpG sites or regions of the *hTERT* gene promoter was seen in the presence of ZnSO_4_ in our study, the results of this study are in line with the results of previous studies, which showed the direct correlation between telomere length, the *hTERT* gene expression, and the telomerase activity.

## Conclusion

This study provides preliminary evidence to support that ZnSO_4_ could decrease the aging of ADSCs via an increase of telomere length, the *hTERT* gene expression, and the telomerase activity, and a decrease in the percentage of senescent cells and the epigenetic modification of the *hTERT* gene promoter. This mentioned effect of ZnSO_4_ at a concentration of 1.5 × 10^−8^ and 2.99 × 10^−10^ M could be used as a good candidate for extending the replicative life-spans of ADSCs in cell therapy and regenerative medicine. Further investigation is required to confirm the data in more samples as well as in protein levels, and it would also be potentially interesting to examine the same project for *in vivo* study.

## Supporting information

S1 Fig Diagram of telomere standard curve. (A) Amplification plots and (B) the corresponding melt curves of the reactions; in (C), the graph shows the standard curve for calculating the length of telomere sequence per reaction tube. (D) Amplification efficiency and R squares of curve. The X-axis represents the number of the cycle and the Y-axis shows the standard’s concentration.
(JPG)

S2 Fig Diagram of a single copy gene (SCG) standard curve. (A) Amplification plots and (B) the corresponding melt curves of the reactions; in (C), the graph shows the standard curve for calculating genome copies using the 36B4 copy number. (D) Amplification efficiency and R squares of curve. The X-axis represents the number of the cycle and the Y-axis shows standard concentrations for each reaction.
(JPG)

S3 Fig Determinate the CpG Islands by the online CpG Islands prediction software. Several CpG islands was shown as light blue color.
(TIF)

S4 Fig A comprehensive genomic view of *hTERT* chromosomal regions was taken by UCSC Genome Browser on Human Dec. 2013 (GRCh38/hg38) Assembly.
(TIF)

RETRACTED

## References

[1] LuW, ZhangY, LiuD, SongyangZ, WanM. Telomeres—structure, function, and regulation. Experimental cell research. 2013;319(2):133–41. doi: 10.1016/j.yexcr.2012.09.005 23006819 PMC4051234

[2] WanTS, MartensUM, PoonSS, TsaoS-W, ChanL, LansdorpPM. Absence or low number of telomere repeats at junctions of dicentric chromosomes. Genes Chromosomes and Cancer. 1999;24(1):83–6. 9892113 10.1002/(sici)1098-2264(199901)24:1<83::aid-gcc12>3.0.co;2-c

[3] Cawthon’s quantitative real-timeP. A quantitative real-time PCR method for absolute telomere length. Biotechniques. 2008;44:807–9. doi: 10.2144/000112761 18476834

[4] BlascoMA. Telomeres and human disease: ageing, cancer and beyond. Nature reviews Genetics. 2005;6(8):611. doi: 10.1038/nrg1656 16136653

[5] WrightWE, ShayJW. Telomere biology in aging and cancer. Journal of the American Geriatrics Society. 2005;53(9s).10.1111/j.1532-5415.2005.53492.x16131355

[6] HiyamaE, HiyamaK. Telomere and telomerase in stem cells. British journal of cancer. 2007;96(7):1020. doi: 10.1038/sj.bjc.6603671 17353922 PMC2360127

[7] ZimmermannS, VossM, KaiserS, KappU, WallerC, MartensU. Lack of telomerase activity in human mesenchymal stem cells. Leukemia. 2003;17(6):1146. doi: 10.1038/sj.leu.2402962 12764382

[8] DevereuxTR, HorikawaI, AnnaCH, AnnabLA, AfshariCA, BarrettJC. DNA methylation analysis of the promoter region of the human telomerase reverse transcriptase (hTERT) gene. Cancer research. 1999;59(24):6087–90. 10626795

[9] GuilleretI, YanP, GrangeF, BraunschweigR, BosmanFT, BenhattarJ. Hypermethylation of the human telomerase catalytic subunit (hTERT) gene correlates with telomerase activity. International journal of cancer. 2002;101(4):335–41. doi: 10.1002/ijc.10593 12209957

[10] NomotoK, MaekawaM, SuganoK, UshiamaM, FukayamaN, FujitaS, et al. Methylation status and expression of human telomerase reverse transcriptase mRNA in relation to hypermethylation of the p16 gene in colorectal cancers as analyzed by bisulfite PCR-SSCP. Japanese journal of clinical oncology. 2002;32(1):3–8. 11932355 10.1093/jjco/hyf001

RETRACTED

[11] BeaneOS, FonsecaVC, CooperLL, KorenG, DarlingEM. Impact of aging on the regenerative properties of bone marrow-, muscle-, and adipose-derived mesenchymal stem/stromal cells. PloS one. 2014;9(12):e115963. doi: 10.1371/journal.pone.0115963 25541697 PMC4277426

[12] Gholizadeh-GhalehazizS, FarahzadiR, FathiE, PashaiaslM. A mini overview of isolation, characterization and application of amniotic fluid stem cells. International journal of stem cells. 2015;8(2):115. doi: 10.15283/ijsc.2015.8.2.115 26634059 PMC4651275

[13] RafiMA. Gene and stem cell therapy: alone or in combination? BioImpacts: BI. 2011;1(4):213. doi: 10.5681/bi.2011.030 23678430 PMC3648974

[14] YuK-R, KangK-S. Aging-related genes in mesenchymal stem cells: a mini-review. Gerontology. 2013;59(6):557–63. doi: 10.1159/000353857 23970150

[15] FathiE, FarahzadiR. Isolation, culturing, characterization and aging of adipose tissue-derived mesenchymal stem cells: a brief overview. Brazilian Archives of Biology and Technology. 2016;59.

[16] LiZ, LiuC, XieZ, SongP, ZhaoRC, GuoL, et al. Epigenetic dysregulation in mesenchymal stem cell aging and spontaneous differentiation. PloS one. 2011;6(6):e20526. doi: 10.1371/journal.pone.0020526 21694780 PMC3111432

[17] AsumdaFZ, ChasePB. Age-related changes in rat bone-marrow mesenchymal stem cell plasticity. BMC cell biology. 2011;12(1):44.21992089 10.1186/1471-2121-12-44PMC3204286

[18] AminizadehN, TiraihiT, Mesbah-NaminSA, TaheriT. Stimulation of cell proliferation by glutathione monoethyl ester in aged bone marrow stromal cells is associated with the assistance of TERT gene expression and telomerase activity. In Vitro Cellular & Developmental Biology-Animal. 2016;52(7):772–81.27251157 10.1007/s11626-016-0021-5

[19] FloresI, CanelaA, VeraE, TejeraA, CotsarelisG, BlascoMA. The longest telomeres: a general signature of adult stem cell compartments. Genes & development. 2008;22(5):654–67.18283121 10.1101/gad.451008PMC2259034

[20] PrasadAS. Zinc: an antioxidant and anti-inflammatory agent: role of zinc in degenerative disorders of aging. Journal of Trace Elements in Medicine and Biology. 2014;28(4):364–71. doi: 10.1016/j.jtemb.2014.07.019 25200490

[21] NemotoK, KondoY, HimenoS, SuzukiY, HaraS, AkimotoM, et al. Modulation of telomerase activity by zinc in human prostatic and renal cancer cells. Biochemical pharmacology. 2000;59(4):401–5. 10644048 10.1016/s0006-2952(99)00334-2

[22] BaoB, AhmadA, AzmiA, LiY, PrasadA, SarkarFH. The biological significance of zinc in inflammation and aging. 2013.

RETRACTED

[23] YusaK, YamamotoO, FukudaM, KoyotaS, KoizumiY, SugiyamaT. In vitro prominent bone regeneration by release zinc ion from Zn-modified implant. Biochemical and biophysical research communications. 2011;412(2):273–8. doi: 10.1016/j.bbrc.2011.07.082 21820411

[24] FathiE, FarahzadiR. Enhancement of osteogenic differentiation of rat adipose tissue-derived mesenchymal stem cells by zinc sulphate under electromagnetic field via the PKA, ERK1/2 and Wnt/β-catenin signaling pathways. PloS one. 2017;12(3):e0173877. doi: 10.1371/journal.pone.0173877 28339498 PMC5365128

[25] FarahzadiR, Mesbah-NaminSA, ZarghamiN, FathiE. L-carnitine effectively induces hTERT gene expression of human adipose tissue-derived mesenchymal stem cells obtained from the aged subjects. International journal of stem cells. 2016;9(1):107. doi: 10.15283/ijsc.2016.9.1.107 27426092 PMC4961110

[26] AmirkhaniMA, MohseniR, SoleimaniM, Shoae-HassaniA, NilforoushzadehMA. A rapid sonication based method for preparation of stromal vascular fraction and mesenchymal stem cells from fat tissue. BioImpacts: BI. 2016;6(2):99. doi: 10.15171/bi.2016.14 27525227 PMC4981255

[27] PirmoradiS, FathiE, FarahzadiR, Pilehvar-SoltanahmadiY, ZarghamiN. Curcumin Affects Adipose Tissue-Derived Mesenchymal Stem Cell Aging Through TERT Gene Expression. Drug Research. 2017.10.1055/s-0043-11963529017189

[28] FathiE, FarahzadiR, RahbarghaziR, KafilHS, YolmehR, editors. Rat adipose-derived mesenchymal stem cells aging reduction by zinc sulfate under extremely low frequency electromagnetic field exposure is associated with increased telomerase reverse transcriptase gene expression. Veterinary Research Forum; 2017: Faculty of Veterinary Medicine, Urmia University, Urmia, Iran.PMC552454428785382

[29] NadriS, SoleimaniM. Comparative analysis of mesenchymal stromal cells from murine bone marrow and amniotic fluid. Cytotherapy. 2007;9(8):729–37. doi: 10.1080/14653240701656061 17917881

[30] AbsalanA, Mesbah-NaminSA, TiraihiT, TaheriT. The effects of cinnamaldehyde and eugenol on human adipose-derived mesenchymal stem cells viability, growth and differentiation: a cheminformatics and in vitro study. Avicenna journal of phytomedicine. 2016;6(6):643. 28078245 PMC5216609

[31] SalehM. The impact of mesenchymal stem cells on differentiation of hematopoietic stem cells. Advanced pharmaceutical bulletin. 2015;5(3):299. doi: 10.15171/apb.2015.042 26504750 PMC4616896

[32] LeviB, JamesAW, NelsonER, VistnesD, WuB, LeeM, et al. Human adipose derived stromal cells heal critical size mouse calvarial defects. PloS one. 2010;5(6):e11177.10.1371/journal.pone.0011177PMC288736120567510

RETRACTED

[33] RakhshandehrooM, HooiveldG, MüllerM, KerstenS. Comparative analysis of gene regulation by the transcription factor PPARα between mouse and human. PloS one. 2009;4(8):e6796. doi: 10.1371/journal.pone.0006796 19710929 PMC2729378

[34] MartinI, JakobM, SchäferD, DickW, SpagnoliG, HebererM. Quantitative analysis of gene expression in human articular cartilage from normal and osteoarthritic joints. Osteoarthritis and Cartilage. 2001;9(2):112–8. doi: 10.1053/joca.2000.0366 11237658

[35] MortazaviY, SheikhsaranF, KhamisipourGK, SoleimaniM, TeimuriA, ShokriS. The evaluation of nerve growth factor over expression on neural lineage specific genes in human mesenchymal stem cells. Cell Journal (Yakhteh). 2016;18(2):189.10.22074/cellj.2016.4313PMC498841727540523

[36] LaiG-J, ShalumonK, ChenJ-P. Response of human mesenchymal stem cells to intrafibrillar nanohydroxyapatite content and extrafibrillar nanohydroxyapatite in biomimetic chitosan/silk fibroin/nanohydroxyapatite nanofibrous membrane scaffolds. International journal of nanomedicine. 2015;10:567. doi: 10.2147/IJN.S73780 25609962 PMC4298333

[37] FathiE, FarahzadiR, CharoudehHN. L-carnitine contributes to enhancement of neurogenesis from mesenchymal stem cells through Wnt/β-catenin and PKA pathway. Experimental Biology and Medicine. 2017;242(5):482–6. doi: 10.1177/1535370216685432 28056548 PMC5367658

[38] MobarakH, FathiE, FarahzadiR, ZarghamiN, JavanmardiS. L-carnitine significantly decreased aging of rat adipose tissue-derived mesenchymal stem cells. Veterinary research communications. 2017;41(1):41–7. doi: 10.1007/s11259-016-9670-9 27943151

[39] Debacq-ChainiauxF, ErusalimskyJD, CampisiJ, ToussaintO. Protocols to detect senescence-associated beta-galactosidase (SA-[beta] gal) activity, a biomarker of senescent cells in culture and in vivo. Nature protocols. 2009;4(12):1798. doi: 10.1038/nprot.2009.191 20010931

[40] BrazvanB, FarahzadiR, MohammadiSM, SahebSM, ShanehbandiD, SchmiedL, et al. Key immune cell cytokines affects the telomere activity of cord blood cells in vitro. Advanced pharmaceutical bulletin. 2016;6(2):153. doi: 10.15171/apb.2016.022 27478776 PMC4961972

[41] O'CallaghanNJ, FenechM. A quantitative PCR method for measuring absolute telomere length. Biological procedures online. 2011;13(1):3.21369534 10.1186/1480-9222-13-3PMC3047434

[42] XiaoC, ZhouH, LiuG, ZhangP, FuY, GuP, et al. Bone marrow stromal cells with a combined expression of BMP-2 and VEGF-165 enhanced bone regeneration. Biomedical Materials. 2011;6(1):015013. doi: 10.1088/1748-6041/6/1/015013 21252414

[43] Noori-ZadehA, Mesbah-NaminSA, Saboor-YaraghiAA. Epigenetic and gene expression alterations of FOXP3 in the T cells of EAE mouse model of multiple sclerosis. Journal of the Neurological Sciences. 2017;375:203–8. doi: 10.1016/j.jns.2017.01.060 28320131

RETRACTED

[44] KatsaraO, MahairaLG, IliopoulouEG, MoustakiA, AntsaklisA, LoutradisD, et al. Effects of donor age, gender, and in vitro cellular aging on the phenotypic, functional, and molecular characteristics of mouse bone marrow-derived mesenchymal stem cells. Stem cells and development. 2011;20(9):1549–61. doi: 10.1089/scd.2010.0280 21204633

[45] EjtehadifarM, ShamsasenjanK, MovassaghpourA, AkbarzadehlalehP, DehdilaniN, AbbasiP, et al. The effect of hypoxia on mesenchymal stem cell biology. Advanced pharmaceutical bulletin. 2015;5(2):141. doi: 10.15171/apb.2015.021 26236651 PMC4517092

[46] BöckerW, YinZ, DrosseI, HaastersF, RossmannO, WiererM, et al. Introducing a single‐cell‐derived human mesenchymal stem cell line expressing hTERT after lentiviral gene transfer. Journal of cellular and molecular medicine. 2008;12(4):1347–59. doi: 10.1111/j.1582-4934.2008.00299.x 18318690 PMC3865677

[47] DesaiN, SabaneghE, KimT, AgarwalA. Free radical theory of aging: implications in male infertility. Urology. 2010;75(1):14–9. doi: 10.1016/j.urology.2009.05.025 19616285

[48] FathiE, FarhzadiR. Survey on impact of trace elements (Cu, Se AND Zn) on veterinary and human mesenchymal stem cells. Rom J Biochem. 2015;52:67–77.

[49] RenL, ZhangA, HuangJ, WangP, WengX, ZhangL, et al. Quaternary ammonium zinc phthalocyanine: Inhibiting telomerase by stabilizing g quadruplexes and inducing g‐quadruplex structure transition and formation. ChemBioChem. 2007;8(7):775–80. doi: 10.1002/cbic.200600554 17361982

[50] LiuQ, WangH, HuD, DingC, XuH, TaoD. Effects of trace elements on the telomere lengths of hepatocytes L-02 and hepatoma cells SMMC-7721. Biological trace element research. 2004;100(3):215–27. doi: 10.1385/BTER:100:3:215 15467107

[51] GuilleretI, BenhattarJ. Unusual distribution of DNA methylation within the hTERT CpG island in tissues and cell lines. Biochemical and biophysical research communications. 2004;325(3):1037–43.10.1016/j.bbrc.2004.10.13715541393

[52] HorikawaI, CablePL, AfshariC, BarrettJC. Cloning and characterization of the promoter region of human telomerase reverse transcriptase gene. Cancer research. 1999;59(4):826–30. 10029071

[53] BryanTM, EnglezouA, Dalla-PozzaL, DunhamMA, ReddelRR. Evidence for an alternative mechanism for maintaining telomere length in human tumors and tumor-derived cell lines. Nature medicine. 1997;3(11):1271–4. 9359704 10.1038/nm1197-1271

[54] BechterOE, EistererW, DlaskaM, KührT, ThalerJ. CpG island methylation of the hTERT promoter is associated with lower telomerase activity in B-cell lymphocytic leukemia. Experimental hematology. 2002;30(1):26–33. 11823034 10.1016/s0301-472x(01)00760-3

RETRACTED

[55] GuilleretI, BenhattarJ. Demethylation of the human telomerase catalytic subunit (hTERT) gene promoter reduced hTERT expression and telomerase activity and shortened telomeres. Experimental cell research. 2003;289(2):326–34. 14499633 10.1016/s0014-4827(03)00281-7

[56] WickM, ZubovD, HagenG. Genomic organization and promoter characterization of the gene encoding the human telomerase reverse transcriptase (hTERT). Gene. 1999;232(1):97–106. 10333526 10.1016/s0378-1119(99)00108-0

[57] TatePH, BirdAP. Effects of DNA methylation on DNA-binding proteins and gene expression. Current opinion in genetics & development. 1993;3(2):226–31.8504247 10.1016/0959-437x(93)90027-m

[58] RamleeMK, WangJ, TohWX, LiS. Transcription regulation of the human telomerase reverse transcriptase (htert) gene. Genes. 2016;7(8):50.27548225 10.3390/genes7080050PMC4999838

[59] RenaudS, LoukinovD, AbdullaevZ, GuilleretI, BosmanF, LobanenkovV, et al. Dual role of DNA methylation inside and outside of CTCF-binding regions in the transcriptional regulation of the telomerase hTERT gene. Nucleic acids research. 2007;35(4):1245–56. doi: 10.1093/nar/gkl1125 17267411 PMC1851636

[60] DengW-G, JayachandranG, WuG, XuK, RothJA, JiL. Tumor-specific activation of human telomerase reverses transcriptase promoter activity by activating enhancer-binding protein-2β in human lung cancer cells. Journal of Biological Chemistry. 2007;282(36):26460–70. doi: 10.1074/jbc.M610579200 17630431

[61] MisitiS, NanniS, FontemaggiG, CongY-S, WenJ, HirteHW, et al. Induction of hTERT expression and telomerase activity by estrogens in human ovary epithelium cells. Molecular and cellular biology. 2000;20(11):3764–71. 10805720 10.1128/mcb.20.11.3764-3771.2000PMC85692

[62] CroweDL, NguyenDC, TsangKJ, KyoS. E2F-1 represses transcription of the human telomerase reverse transcriptase gene. Nucleic Acids Research. 2001;29(13):2789–94. 11433024 10.1093/nar/29.13.2789PMC55771

[63] GoueliBS, JanknechtR. Regulation of telomerase reverse transcriptase gene activity by upstream stimulatory factor. Oncogene. 2003;22(39):8042–7. doi: 10.1038/sj.onc.1206847 12970752

